# Physical Activity Level and Social-Ecological Influence Factors in Chinese Information Technology Professionals: A Cross-Sectional Study

**DOI:** 10.1155/2022/4580589

**Published:** 2022-08-26

**Authors:** Lejun Wang, Hua Yang, Xiaoqian Song, Ce Wang, Minjie Qiao, Haifeng Tao, Wenxin Niu, Ruijie Li

**Affiliations:** ^1^Sport and Health Research Center, Physical Education Department, Tongji University, Shanghai 200092, China; ^2^Shaanxi Institute of Sports Science, No. 303 Zhangba East Road, Xi'an 710065, Shaanxi, China; ^3^Shanghai Yangzhi Rehabilitation Hospital, School of Medicine, Tongji University, Shanghai 201619, China

## Abstract

**Objective:**

Information technology (IT) population in China has expanded rapidly in recent decades, which has suffered severe health problems due to a lack of physical activity (PA). However, little is known about the influence and solutions of PA deficiency. The current research was designed to explore the associations between the amount of PA and potential influenced factors based on the social-ecological model (SEM) and thus to provide rationales for PA promotion.

**Method:**

Six hundred and five IT professionals from five cities of China were surveyed in terms of PA in daily life as well as the potential PA influence factors based on SEM models that consisted of individual, interpersonal, environmental, and political levels in the current study. Hierarchical linear regression analyses were conducted to examine the association of the potential PA influence factors and PA amount.

**Result:**

About 54.7% of the sample did not fulfill the PA recommendation of 600 MET per week, and there are significant gender differences in PA participation. Factors related to the individual (self-efficacy and value recognition), interpersonal (social support), environmental (workplace and community environment), and polity-level factors (policy advocacy) were found to be significantly associated with Chinese IT professionals' participation in PA.

**Conclusion:**

Numerous correlates from individual-level to political-level factors are all important predictors of PA. Exercise value recognition and self-efficacy accounted for much of the association. Environmental variables may further influence exercise behavior. Therefore, conducting intervention efforts for individual, interpersonal, environmental, and political change of Chinese IT professionals is recommended.

## 1. Introduction

In the past decade in China, the industry of information technology (IT) has witnessed a great expansion with a compound annual growth rate of more than 8% [1]. The rapid development of the IT industry induced a sharp increase in IT employees. In 2019, the number of IT employees was 9.11 million, which is expected to increase by about 306,000 per year in the following 20 years of China [2]. However, the IT population in China has been characterized by long time concentration working hours, staying up late, bearing great stress, and serious sedentary behavior in daily life due to the fierce industry competition as well as the need for high technical professionalism, which is different from other nonmanual labors and has contributed to severe health problems in the IT population [3–5]. As a result, the IT population in China has suffered a high incidence of many diseases and even sudden cardiac death (SCD), which remains an important public health issue accounting for an estimated incidence rate (41.8 of 100,000 per year) [6, 7]. It has been presumed that the approximate annual incidence of SCD among the 9.11 million IT employees is about 4,000.

Exercise is the best medicine. Regular physical activity (PA) can greatly improve physical fitness and reduce the incidence risk of many diseases. In previous researches, sedentary behavior and lack of regular exercise have been explained for the incidence of many diseases [8, 9]. As the “996” work system (9 a.m. to 9 p.m., 6 days a week) became a corporate culture, especially in Chinese high-tech industries in recent years, it has been adopted by many famous IT enterprises such as Alibaba, Tencent, Jingdong, and so on [10]. As a result, a substantial proportion of the professionals are apt to stay sedentary to work for more than 9 hours per day without regular PA and sufficient sleep. Therefore, it is urgent to promote the physical activities of IT populations in China to reduce health problems and relieve the social burden on medical treatment.

In early relevant researches, intrapersonal factors (i.e., characteristics and motivation of the individual) have been concerned and recognized as the key factor to determine the PA [11]. In the later studies, other factors such as interpersonal, environmental, communal factors, and public policy have also been researched and proved to be influential in PA [12–14]. However, both intrapersonal and other factors have rarely been fully considered in the researches of PA promotion until the adoption of social-ecological models (SEM). SEM suggests that there are multiple interacting layers that influence PA behavior [15]. While SEM has been wildly used in the field of PA promotion in adults around the world [16, 17], However, little is known about the influence factors and promotion way of PA in the Chinese IT population.

Based on the above researches, we hypothesize that the PA of IT employees may be closely related to the factors of the SEM. The current research was designed to verify the hypothesis and thus provide a rationale for PA promotion among IT populations.

## 2. Methods

### 2.1. Study Design and Participants

This study was conducted to acquire the amount of physical activities and their influence factors on IT professionals in China. A questionnaire was designed and applied to investigate the issue. Data collection was conducted via a network questionnaire survey platform (https://www.wjx.cn/) between September and October of 2020. Stratified sampling was employed considering companies' ownership, size, location, and industrial status to recruit 605 participants in 5 high-developed IT industry cities (Beijing, Shanghai, Dalian, Hangzhou, and Shenzhen) in China. The inclusion criteria of participants were: (1) IT professionals including programmers, system analysts, web developers, test engineers, as well as IT managers; (2) more than 1 year of working experience in the IT industry; (3) age 20 to 60 years, (4) healthy with no psychological disorders or mental problems, (5) having no history of using drugs, narcotics, and substances; and (6) volunteered to participate in this survey. Before the formal questionnaire, informed written consent was obtained from all participants. The study received ethical approval from the Ethics Committee of Tongji University of Medical Sciences.

### 2.2. Instrument

PA and its potential determinants were intended to acquire use an ad hoc self-administered questionnaire based on the survey of our target population. The questionnaire included three parts. The first part of the questionnaire was designed to collect information including age, gender, weight, height, socioeconomic level, marital status, educational level, work experience, and self-perception of the health status. In the second part, participants self-reported the frequency and duration of walking, transport-related PA, leisure-time PA, and sitting time in a typical week. The third section was applied to survey the potential PA influence factors based on SEM that consisted of individual, interpersonal, environmental, and political levels in the current study. In order to improve the reliability of the survey results, parallel questions were designed in the questionnaire. All variables of the SEM instrument were measured using a five-point Likert scale, ranging from 1 (strongly disagree) to 5 (strongly agree). For variables with more than one item, items were summed to calculate a total score for that variable [18].

#### 2.2.1. PA

The amount of physical activity of each participant was calculated based on the survey data on frequency and duration of walking, transport-related physical activity, leisure-time physical activity, and sitting time of subjects in a typical week. According to previous research [19], we divided the physical activity of the respondents into three levels: light-intensity PA (LPA), moderate-intensity PA (MPA), and vigorous-intensity PA (VPA) [20]. The metabolic equivalent (MET) was used to weight each type of PA by its energy expenditure, with 8 METs for VPA, 4 METs for MPA, 3.3 METs for LPA, and 1 MET for sedentary activity [21, 22]. Based on the weighted calculations, we defined LPA as less than 600 MET mins·wk.^− 1^, MPA as a practice between 600 and 1,500 mins·wk.^− 1^, and VPA as more than 1,500 mins·wk.^− 1^ [9, 23]. The weight of each activity intensity was derived from the international physical activity questionnaire (IPAQ) scoring protocol [19]. Based on the physical activity guidelines recommended by WHO and the American College of Sports Medicine (ACSM) for healthy adults, the participants' results were assessed to determine whether they were getting sufficient exercise (i.e., 150 min moderate exercise per week) [24].

#### 2.2.2. Individual Variables

Self-efficacy related to PA was self-reported by IT professionals on the survey using a tested scale consisting of seven items that gauged subjects' confidence and recognition in their ability to overcome barriers and to be active. The content showed a high internal consistency (*α* = 0.927). Value recognition regarding participation in PA was assessed with four items. Example items include “exercise is troublesome, and I do not like it”; “lack of company and find it boring to exercise alone”; and so on. The internal consistency of this scale was 0.839.

#### 2.2.3. Interpersonal Variables

Perceived support from family members and peers were each self-reported by subjects on the PA survey using four items for each scale. IT professionals indicated how often their family or one of their friends provided support related to PA during a typical week and include responses such as “encouraged or advised you to do physical activities” and “accompany you to participate.” Construct reliability (CR) and average variance extracted (AVE) values for these scales were 0.867 and 0.700, respectively, and the alpha Cronbach's coefficient was 0.84. The higher the score on scales indicated the higher levels of social support among participants.

#### 2.2.4. Environmental Variables

The company and community PA environment were evaluated via newly developed validated self-reported scales with nine items. For example, “there are multiple fitness venues around your company or community.” The internal consistency for this scale was *α* = 0.935. The facility environment was measured using a four-item scale. All responses capture the availability and accessibility of equipment and other resources that may support participation in PA. An example question was “Facilities in your community can meet your sporting needs.” Reliability for the infrastructure quality scale was *α* = 0.868 in this sample.

#### 2.2.5. Political Variables

Political variables are proposed to access the impact of public policies and social media promotion on PA. The sample items acquire whether subjects have ever watched various TV and Internet programs or participated in various sports activities organized by government departments and social organizations. A score indicating the total number of political advocacies was created by summing the responses to each item. CR and AVE values for the scale were 0.864 and 0.796, respectively; the alpha Cronbach's coefficient was 0.86.

### 2.3. Statistics Analysis

Statistical analysis was performed using IBM SPSS 25.0 (SPSS Inc., Chicago, IL). Cronbach's alpha test was conducted to assess the internal consistency of the instrument, with a value over 0.8, indicating favorable reliability. Spearman cross-correlation analysis was used to determine the parallel-test reliability of the survey. The chi-square test was used to determine the difference between different sociodemographic variables and levels of PA. One-way analysis of variance (ANOVA) was adopted to test the within-group variation between the score of varied subscale and the PA levels. Spearman correlation matrix was computed and reproduced to see the bivariate relationships between proposed SEM predictors and outcome variables. In the end, hierarchical linear regression analyses were conducted to examine the association of the individual, interpersonal, environmental, and polity subscales with attaining the recommended level of PA, 95% confidence intervals were calculated for each variable. Meanwhile, we examined the beta coefficients for each outcome predicting PA levels as well as model fit based on *R*^2^ and change in *R*^2^ (Δ*R* [2]) per step of the model. All significance thresholds were set at *α* = 0.05.

## 3. Results

### 3.1. Basic Characteristics of the Respondents

A total of 605 Chinese IT professionals aged 18 to 60 years with a BMI of 24.37 ± 11.57 kg/m^2^ completed the study. The characteristics of the participants are shown in Table 1. The participants consisted of 63.8% males and 36.2% females. A total of 81.7% of the participants were younger than 46 years old. A total of 45.45% of subjects were unmarried, while 0.66% of subjects were divorced. Besides, the numbers of participants with an associate degree, bachelor's degree, postgraduate degree, and doctoral degree were 90 (14.88%), 342 (56.53%), 141 (23.31%), and 21 (3.47%), respectively. A total of 92.1% of the participants (557 of 605) had total years of work experience of less than 15 years.

### 3.2. Association between Demographic Variables and the Level of PA

The results (Table 1) showed that 45.3% of the respondents attained the recommended level of PA (≥600 MET·wk.^–1^) and males are more likely to reach the recommended level than females (*χ*2 = 21.581, *P* < 0.001). Meanwhile, married IT professionals were significantly more inactive in PA than unmarried individuals (*χ*2 = 18.112, *P* < 0.001). On the other hand, most of our participants had higher education, and the rate of PA was significantly higher among people with a diploma than the others (*χ*2 = 21.850, *P* < 0.01).

The descriptive statistics of SEM factors in individuals, interpersonal level, and environmental level are shown in Table 2. The energy expenditure of the spontaneous PA of the whole participants is 788.30 ± 609.16 MET mins·wk.^–1^. The self-efficacy variable (28.32 ± 5.95) at the individual level is higher than other factors, followed by workplace and community environment factors (27.41 ± 8.46) at the environmental level, and the policy level (5.62 ± 2.23) is the lowest. Participants engaging in more than 600 MET mins·wk.^–1^ of PA energy expenditure are higher in the subscales for self-efficacy and value recognition. In contrast, the lower PA individuals had less social support.

Spearman correlation coefficient between all variables of SEM constructs and PA level is shown in Table 3. Among all variables, self-efficacy (*r* = 0.23), value recognition (*r* = 0.25), social support (*r* = 0.18), workplace and community environment (*r* = 0.16), and political advocacy (*r* = 0.21) were significantly, positively associated with PA level (all *P* < 0.001). We also found that higher self-efficacy scores were significantly associated with social support (*r* = 0.46), political advocacy (*r* = 0.31), and workplace/community environment (*r* = 0.28) factors other than value recognition (*r* = 0.03). Conversely, a higher value recognition score was associated with more facility environment factors (*r* = 0.54) compared to other variables. Social support scores were significantly associated with all variables, especially with the workplace/community environment factors (*r* = 0.52). There was a strong positive association between having a more active environment in the workplace or community and vigorous public political advocacy (*r* = 0.59).

In the hierarchical logistic regression model (Table 4), step 1 assesses the influence of individual-level (self-efficacy and value recognition) on PA. The results showed that individual variables explained a statistically significant 8% of the PA. Step 2 including the social support variable added significantly to the model. In this step, the predictive effect of the individual and interpersonal levels was investigated, and the results showed that the factors predict up to 8.9% of PA. In step 3, the predictive effects of individual, interpersonal, and environmental factors were examined, and the results showed that these variables predicted about 10.7% of PA. In step 4, the addition of political advocacy variables added a significant additional 0.7% variance explaining PA. Overall, the model explained 11.2% of the variance in PA levels.

## 4. Discussion

This study aimed to determine individual, interpersonal, environmental, and political predictors of PA consumption among Chinese IT professionals. Results from this study indicate that the pattern of bivariate correlations among SEM variables and PA level differed in magnitude from political level to individual-level factors. To our knowledge, it is the first time to explore the influence factors of physical activities based on the social-ecological framework in Chinese IT populations.

In this study, it was found that 54.7% of Chinese IT professionals are not meeting the recommended 600 MET of weekly PA consumption, which is consistent with previous studies in a large cohort of younger to middle-aged adults [20]. As numerous Chinese Internet companies have adopted the “996” working hour system as their official work schedule, it is reasonable to find that working for 9–12 h per day is common in high-tech industrial enterprises [10]. Results from previous studies examining the integration of PA into daily work life, especially for those in sedentary occupations, can have a considerable impact on reducing the burden of preventable overweight and its related diseases [25]. Moreover, education, marital, and health status are most closely related to the PA of Chinese IT professionals. Our study also found the existence of important gender differences in the level of PA among participants. Males report higher levels of sedentary behavior than females, while females less frequently reach WHO recommended levels of PA than males. Gender differences may be attributed to differences in occupational or social roles [25].

Health behaviors are shaped through a complex interplay of determinants at various levels, and social-ecological models suggest that these multiple levels of influence interact across levels [26]. This study found obvious evidence of an association between individual, interpersonal, environmental, and political variables and different PA levels among IT professionals. The results of this study were consistent with the SEM tenets, which provide support for our initial hypothesis that various theoretical factors underlying individual, interpersonal, environmental resources, and political factors are associated with IT professionals' participation in PA.

It should be noted that individual factors were found to be direct predictors of PA, with value recognition even stronger than self-efficacy [27, 28]. The analyses of the relationship between subjects' individual scale scores and PA levels indicated that most Chinese IT professionals tend to put more effort to engage in PA. It is also worth highlighting that the variables at the individual level not only accumulated the highest average score but also contributed to the most variance explanation rate of PA engagement. As a central determinant of social cognitive theory, self-efficacy was the direct influence factor exerted by the participants' beliefs in their ability to be physically active [29, 30]. Besides, the results demonstrated that value recognition had a higher relationship with PA than intentions, which may be related to the personal knowledge, attitudes, beliefs, and motivation in initiating and maintaining PA [31]. Our study also demonstrated that a higher PA level was accompanied by a higher level of education among IT professionals. However, although the intention is a necessary factor for a person to be physically active, a wide range of barriers across the four social-ecological levels may also prevent the participation of PA [32].

Interpersonal factors appear to be potentially important since they demonstrated associations with more active PA participation. As a representative variable, social support for exercise from family members, friends, and colleagues is probably the most clearly confirmed determinant. Similar to another study [33], our results showed that social support had a high correlation with exercise self-efficacy score (*r* = 0.458) and interpersonal variables may likely affect PA indirectly through one's perception of exercise self-efficacy and value recognition [31]. Besides, some studies have indicated that coworker social support is an important correlate of PA for office workers [34]. Although adult employees are likely to have more leisure time exposure with family members, workplace support is an important setting for health promotion, and employee behavior is largely influenced by coworker health-related norms and values [35, 36]. Hence, the results suggest that employees may benefit from greater visibility for positive PA behaviors, perhaps through interpersonal or workplace support.

Among the rapidly increasing number of international research studies, environmental factors are thought to have widespread effects on PA [37]. Workplace and community-level factors were shown to be important regarding PA participation among Chinese IT professionals. Our findings confirmed previous research suggests that facility environment (i.e., exercise equipment at the company, access to facilities) and community-level influences such as enjoyable scenery, owner activities, and frequent observation of others engaging in PA may be significant correlates [38]. Environmental factors may influence constraints on behavior and perceptions making it easier or more difficult to participate in PA [39]. Remarkably, as the workplace became an important area for health campaigns of many kinds as well as basic occupational health, employers must pay more attention and invest in the health of their employees to reduce sickness absence, increase productivity, and better staff retention [40]. The influence of the environmental factors on participation remains a high-priority area for future research [41].

Finally, the positive relationships between the political factors and PA participation deserve mention. The development and implementation of national policies may contribute to the creation of supportive environments for people to engage in physically active lifestyles [42]. Our findings revealed that policy factors contributed to predicting the PA behavior of Chinese IT professionals, while participants have a lower average score at the policy level compared with other indicators. This may be related to the absence of national PA guidelines as well as necessary monitoring systems of implementation. Although the Chinese government has introduced some policies and actions (e.g., Healthy China 2030 Blueprint) to minimize the health burden and encourage people to actively engage in physical activities [43], PA promotion is an intersectoral challenge, and it also needs a coordinated approach to policy development and implementation across all levels of government to ensure complementary policy action [44]. To this end, more research initiatives are warranted to address the present paucity of knowledge regarding the policy-level factors, as well as their direct and indirect effects on participants' engagement in PA [45].

However, limitations should be also acknowledged in the current study. First, it would be argued that the results of the current study could be influenced by the COVID-19 pandemic as all working staff were asked to work at home since February 2020, which may significantly influence all people's participation in PA. However, due to the effective solutions to the COVID-19 pandemic, normal work and lifestyles have recovered since April 2020 in China, which may greatly reduce the influence of the COVID-19 pandemic and indicate the rationale of the current results. Second, it would be better to expand the sample size to increase the statistical power due to the large number of IT populations in China. Third, the limitations of gender effect on the results as the number of male and female participants are distinct in the current study. Despite the limitations above, SEM has been firstly adopted to explore the PA of Chinese IT professionals, which may at least give insights into PA promotion among IT populations.

## 5. Conclusions

Numerous correlates from individual-level to political-level factors are all important predictors of PA. Exercise value recognition and self-efficacy accounted for much of the association. Environmental variables may further influence exercise behavior. Therefore, conducting intervention efforts for individual, interpersonal, environmental, and political change of Chinese IT professionals is recommended.

## Figures and Tables

**Table 1:** Demographic characteristics of participants, by PA.

Variables	PA level			*N*	%	*χ*2	*P*
	LPA	MPA	VPA				
Gender						21.581	*P* ≤ 0.001
Male	189	136	61	386	63.80%		
Female	142	65	12	219	36.20%		

Age (year)						2.489	*P*=0.870
≤25	51	33	13	97	16.03%		
26–35	185	104	39	328	54.21%		
36–45	89	57	20	166	27.44%		
46–60	6	7	1	14	2.31%		

Education						21.850	*P* ≤ 0.01
Doctoral degree	7	8	6	21	3.47%		
Master's degree	59	59	23	141	23.31%		
Bachelor's degree	207	102	33	342	56.53%		
Associate degree	51	30	9	90	14.88%		
HS graduate/less than HS	7	2	2	11	1.82%		
Marital status						18.112	*P* ≤ 0.001
Single, never married	127	114	34	275	45.45%		
Married	201	86	39	326	53.88%		
Separated/divorced	3	1	0	4	0.66%		

Income (RMB/YEAR)						12.555	*P*=0.128
≤100,000	113	56	19	188	31.07%		
100,000–200,000	102	54	20	176	29.09%		
200000–300000	55	33	11	99	16.36%		
300,000–400,000	23	23	6	52	8.60%		
＞400,000	38	35	17	90	14.88%		

Work experience						2.831	*P*=0.945
＜3 years	94	63	20	177	29.26%		
3–6 year (exclude 6 years)	71	40	19	130	21.49%		
6–10 years (exclude 10 years)	72	38	14	124	20.50%		
10–15 years (exclude 15 years)	70	41	15	126	20.83%		
≥15 years	24	19	5	48	7.93%		

Perceived health						37.904	*P* ≤ 0.001
Very good	14	21	18	53	8.76%		
Rather good	107	75	30	212	35.04%		
Subhealth	187	91	23	301	49.75%		
Rather poor	21	13	2	36	5.95%		
Very poor	2	1	0	3	0.50%		

LPA: light PA, MPA: moderate PA, and VPA: vigorous PA. Notes: ^*∗*^*P*=<0.05, ^*∗∗*^*P*=<0.001, and ^*∗∗∗*^*P*=<0.0001.

**Table 2:** Descriptive statistics of SEM factors and PA levels among subjects, by PA level (*N* = 605).

Variable	Mean ± SD	PA level			*F* ^a^	*P* value
		LPA	MPA	VPA		
PA level	788.30 ± 609.16	405.49 ± 96.43	932.16 ± 250.42	2127.98 ± 587.32	2,551.905	*P* ≤ 0.001

Individual level						
Self-efficacy	28.32 ± 5.95	27.11 ± 6.30	29.46 ± 5.02	30.67 ± 5.39	33.144	*P* ≤ 0.001
Value recognition	11.50 ± 4.07	10.74 ± 3.27	12.13 ± 4.49	13.25 ± 5.12	31.256	*P* ≤ 0.001

Interpersonal level						
Social support	13.36 ± 3.46	12.84 ± 3.01	14.04 ± 3.59	13.80 ± 4.25	12.082	*P* ≤ 0.001

Environment level						
Facility environment	11.12 ± 4.07	11.19 ± 3.83	11.21 ± 4.00	10.56 ± 5.16	0.812	*P*=0.368
Workplace/community environment	27.41 ± 8.46	26.19 ± 7.78	28.80 ± 8.67	29.12 ± 9.92	13.627	*P* ≤ 0.001

Political level						
Political advocacy	5.62 ± 2.23	5.22 ± 2.10	6.12 ± 2.19	6.08 ± 2.51	20.182	*P* ≤ 0.001

LPA: light PA, MPA: moderate PA, and VPA: vigorous PA. ^a^Using the analysis of variance. ^*∗∗*^*P* < =001 and ^*∗∗∗*^*P* < 0.0001.

**Table 3:** Spearman Correlations between PA level and SEM constructs (*N* = 605).

Variable	PA level	SEM constructs					
		SE	VR	SS	FE	WE/CE	PA
PA level	1						
Self-efficacy	0.233^*∗∗∗*^	1					
Value recognition	0.248^*∗∗∗*^	0.035	1				
Social support	0.177^*∗∗∗*^	0.458^*∗∗∗*^	−0.215^*∗∗∗*^	1			
Facility environment	−0.034	−0.257^*∗∗∗*^	0.541^*∗∗∗*^	-0.367^*∗∗∗*^	1		
Workplace/community environment	0.159^*∗∗∗*^	0.277^*∗∗∗*^	−0.174^*∗∗∗*^	0.521^*∗∗∗*^	−0.249^*∗∗∗*^	1	
Political advocacy	0.210^*∗∗∗*^	0.307^*∗∗∗*^	−0.112^*∗∗∗*^	0.478^*∗∗∗*^	−0.295^*∗∗∗*^	0.590^*∗∗∗*^	1

SE: self-efficacy, VR: value recognition, SS: social support, FE: facility environment, WE/CE: workplace/community environment, and PA: political advocacy. Note.^*∗∗∗*^*P* < 0.0001.

**Table 4:** Results of hierarchical regression analyses explaining PA-related factors according to SEM.

Step/predictor variable	*R* ^2^ (adjusted)	Δ*R*^2^ (adjusted)	Beta^a^	95% CI		*F*	*P* value
				Lower	Upper		
Step 1: individual level	0.08	0.083	—	—	—	27.296	*P* ≤ 0.001
Self-efficacy	—	—	0.118	3.062	21.082	—	—
Value recognition	—	—	0.295	30.033	58.588	—	—
Step 2: interpersonal level	0.089	0.010	—	—	—	20.635	*P* ≤ 0.001
Social support	—-	—	0.015	−15.683	20.871		
Step 3: environment level	0.107	0.021	—	—	—	15.454	*P* ≤ 0.001
Facility environment	—	—	−0.13	−34.456	-4.518	—	—
Workplace/community environment	—	—	0.061	−3.219	11.977	—	—
Step 4: political level	0.112	0.007	—	—	—	13.702	*P* ≤ 0.001
Political advocacy	—	—	0.109	2.186	57.325	—	—

^a^Standardized regression coefficients.

## Data Availability

The raw data supporting the conclusions of this article will be made available by the authors, without undue reservation.

## Abbreviations

PA: Physical activity
IT: Information technology
SCD: Sudden cardiac death
SEM: Social-ecological model
MET: Metabolic equivalent
LPA: Light-intensity physical activity
MPA: Moderate-intensity physical activity
VPA: Vigorous-intensity physical activity
IPAQ: International physical activity questionnaire
WHO: World Health Organization
ACSM: American College of Sports Medicine
CR: Construct reliability
AVE: Average variance extracted
ANOVA: Analysis of variance.
